# A Pulmonary Vascular Extraction Algorithm from Chest CT/CTA Images

**DOI:** 10.1155/2021/5763177

**Published:** 2021-11-05

**Authors:** Shihui Xu, Ziming Zhang, Qinghua Zhou, Wei Shao, Wenjun Tan

**Affiliations:** ^1^Key Laboratory of Intelligent Computing in Medical Image, Ministry of Education, Shenyang 110189, China; ^2^College of Computer Science and Engineering, Northeastern University, Shenyang 110189, China

## Abstract

Segmentation of pulmonary vessels in CT/CTA images can help physicians better determine the patient's condition and treatment. However, due to the complexity of CT images, existing methods have limitations in the segmentation of pulmonary vessels. In this paper, a method based on the separation of pulmonary vessels in CT/CTA images is investigated. The method is divided into two steps: in the first step, the lung parenchyma is extracted using the Unet++ algorithm, which can effectively reduce the oversegmentation rate; in the second step, the pulmonary vessels in the lung parenchyma are extracted using nnUnet. According to the obtained lung parenchyma segmentation results, the “AND” operation is performed on the original image and the lung parenchyma segmentation results, and only the blood vessels within the lung parenchyma are segmented, which reduces the interference of external tissues and improves the segmentation accuracy. The experimental data source used CT/CTA images acquired from the partner hospital. After the experiments were performed on a total of 67 sets of images, the accuracy of CT and CTA images reached 85.1% and 87.7%, respectively. The comparison of whether to segment the lung parenchyma and with other conventional methods was also performed, and the experimental results showed that the algorithm in this paper has high accuracy.

## 1. Introduction

With the development of 5G technology, the high speed and stability of 5G networks can provide new platforms and ideas for remote diagnosis and treatment. 5G networks can transmit massive image data files quickly and reliably, which requires more accurate image processing algorithms to match them. As a major category of diseases affecting human health, the processing of lung images has been the focus of various types of research. Lung tissue extraction is used as a prerequisite for remote image diagnosis and treatment, and a more accurate algorithm for lung vessel segmentation will be investigated in this paper.

Currently, surgery for the lung requires clinicians to have more experience and information about the patient itself to determine a more accurate scope of surgery, but it takes a long time for clinicians to train and grow in experience, so it is important to provide clinicians with more valid information about the patient's condition. With the continuous development of CT scanning technology, the patient information displayed in chest CT is becoming clearer and clearer, which enables doctors to get more and more detailed information, so how to provide doctors with more accurate and objective information about the preoperative tissue structure localization and cancerous lesions is an urgent problem in clinical application [1, 2].

The analysis of medical images first requires image processing, which helps to highlight key information in the images, so the development of medical image processing is crucial. Currently, medical image segmentation algorithms are mainly divided into traditional methods and deep learning-based algorithms. Among them, traditional methods mainly include methods based on threshold [3], edges, regions, and morphology. Deep learning-based algorithms are mainly based on convolutional neural networks [4–6] or their improvement methods [7–9].

Segmentation of pulmonary parenchyma is a fundamental task in chest CT image segmentation processing, which can be used as a prework for pulmonary vascular and segmentation. Jin et al. [10] has proposed an easy-to-implement pulmonary parenchyma segmentation algorithm for chest CT images with the presence of borderline pulmonary nodules by integrating an improved two-dimensional convex packet algorithm with region growth and morphology for pulmonary contour and internal structure. Chen et al. [11] proposed a dense deep convolutional network (LDDNet) for the pulmonary, which used some common optimizer methods such as dense block, batch normalization, and undersampling operations. Xiao et al. [12] combined the threshold iterative segmentation method with the fractal geometry method for detecting the pulmonary depression boundary to perform the initial segmentation of the pulmonary parenchyma and then completed the accurate segmentation of the pulmonary parenchyma by convex packet repair to complete the accurate segmentation of pulmonary parenchyma. Raj et al. [13] used active contours with the distance regularization level set method to perform automatic segmentation of pulmonary parenchyma regions, avoiding the repetition of initialization again. Yoo et al. [14] performed the training of pulmonary parenchyma segmentation models using two-dimensional Unet and three-dimensional Unet networks and then segmented the left and right lungs separately.

For the segmentation of pulmonary vessels, there are mainly fast marching methods, vessel enhancement filter method, and wavefront propagation-based methods [15]. Yang et al. used multiscale filters for different sizes of blood vessels to perform extraction of maximum response scale information and then extracted blood vessels by dynamic threshold. Hao Jutao et al. performed blood vessel segmentation based on the fuzzy clustering algorithm. Zhou et al. [16] proposed a pulmonary blood vessel segmentation algorithm based on expectation maximization analysis and morphological knowledge, firstly, through a three-dimensional multiscale filtering algorithm. The enhancement of vascular voxels was performed while suppressing other structures, and then, high response voxels were extracted and expectation maximization was used to segment the obtained pulmonary vessels. Orkisz et al. [17] proposed a pulmonary vessel extraction method based on Hessian matrix that can be calculated automatically according to the actual situation changes.

In this paper, the theory of deep learning-based pulmonary vascular segmentation algorithm in CT chest imaging will be thoroughly investigated, expecting to provide thoracic surgeon clinicians and imaging physicians with an accurate and objective algorithm based on conventional CT image analysis for the preoperative separation of pulmonary vessels belonging to target segments in thoracoscopic lung segment resections in a fully automated manner. This paper combines lung parenchymal segmentation with pulmonary vascular segmentation to improve the accuracy of pulmonary vascular segmentation.

## 2. Materials and Methods

This paper is divided into two parts: firstly, the segmentation of the lung parenchyma and then the segmentation of the pulmonary vasculature based on this, in which the lung parenchyma segmentation part uses the Unet++ network to segment the lung parenchyma, and the obtained lung parenchyma part, which removes other tissues outside the lung parenchyma range. The pulmonary vascular segmentation part implements a pulmonary vascular segmentation algorithm based on the nnUnet network, which directly segments the vasculature inside the lung parenchyma and reduces the interference of irrelevant tissues in the extrapulmonary region.

### 2.1. Lung Parenchyma Segmentation Based on the Unet++ Network

The Unet++ network [18] is based on the Unet network with improvements, which is still essentially an encoder-decoder structure based on deep supervision. But it also differs from the Unet network in many ways by redesigning more dense jump connections, narrowing the semantic gap between encoded and decoded subnetwork feature mappings and making the network more sensitive to fine-grained target structures.

In the Unet network, a jump connection is adopted for feature fusion, which fuses fine-grained features in the encoder with coarse-grained features in the decoder to help the decoder recover finer semantic details of the target part more efficiently during upsampling. Unet++ retains the feature fusion in Unet and adds short connections between Unet networks of different depths as a way to retain more image information from the upper layer of operations.

The network structure of the Unet++-based lung parenchyma segmentation algorithm implemented in this paper is as follows. Firstly, the original image is downsampled, and the downsampling operation can reduce the influence of some disturbances on the input image, decrease the amount of network operations, increase the size of the training perceptual field, and reduce the probability of overfitting of the results. Jump connections and long connections are used to transfer information between the same layers. Finally, the result of each layer is upsampled, and the previously extracted image features are decoded and reduced to the size of the original image, which is fused using the fusion layer, and finally the segmentation result is obtained.

In the network training process, the input data are PNG images, where the size of the 2D images of each data set is 512 × 512, the batch size is set to 2, 150 epochs are trained, the activation function is used as the ReLU function in equation (1), and the loss function is used as the sum of the DICE coefficients and the cross-entropy loss function in equation (2), where *X* is the labeled good image and *Y* is the predicted segmentation result. |*X*∩*Y*| denotes the number of pixels in the intersection of *X* and *Y*, and |*X*+*Y*| denotes the sum of the number of pixels in *X* and *Y*. The initial learning rate is 0.0001.

(1) ReLu=max0,x,lossX,Y=−1n∑i=1n12X  log  Y+2X∩YX+Y.

The optimizer uses the Adam function in equation (3):

(2) $$\begin{array}{c} \theta_{t+1}=\theta_{t}-\frac{\eta }{\sqrt{{\tilde{v}}_{t}+\varepsilon }}{\tilde{m}}_{t}, \end{array}$$

where *η* denotes the learning rate and *ε* denotes the minimal value that maintains the stability of the numerical computation. ${\tilde{m}}_{t}$ and ${\tilde{v}}_{t}$ denote the first-order moment estimate and second-order moment estimate of the gradient, respectively, which are calculated as follows:

(3) $$\begin{array}{c} {\tilde{m}}_{t}=\frac{m_{t}}{1-\beta_{1}^{t}},\\ {\tilde{v}}_{t}=\frac{v_{t}}{1-\beta_{2}^{t}}, \end{array}$$

where ${\tilde{m}}_{t}$ and ${\tilde{v}}_{t}$ are calculated as follows:

(4) $$\begin{array}{c} m_{t}=\beta_{1}m_{t-1}+\left(1-\beta_{1}\right)g_{t},\\ v_{t}=\beta_{2}v_{t-1}+\left(1-\beta_{2}\right)g_{t}^{2}. \end{array}$$

### 2.2. Pulmonary Vascular Extraction Based on nnUnet++ Network from Parenchyma Region

nnUnet [19, 20] is a framework proposed based on the Unet network, which is based on the original Unet network and does not make new changes to the network structure, but combines three structures, 2D Unet, 3D Unet, and Unet cascade, which can adapt to different datasets and automatically select a more suitable network to complete the segmentation task. Focusing the image segmentation task on image preprocessing, training inference, and image postprocessing, overfitting of segmentation results is avoided due to the complexity of the network.

The nnUnet network structure contains three main parts: 2D Unet, 3D Unet, and Unet cascade. The left half of 2D Unet is the encoding part. 3D Unet has the same structure as 2D Unet as a whole, except that the 2D operation is converted to 3D. The Unet cascade structure is used to solve the problem of the large amount of data needed for the 3D Unet network.

The network structure of the nnUnet-based pulmonary vascular segmentation algorithm implemented in this paper is shown in Figure 1. The segmentation of pulmonary vessels is performed using a 3D Unet cascade structure, where data are first preprocessed by resampling and normalization, then the coarse segmentation of the pulmonary vessel part is performed by the first 3D Unet, and the results are integrated with the original data before the target is performed by the second 3D Unet refinement segmentation to obtain the final results.

The pulmonary vascular segmentation network is trained by combining the lung parenchyma segmentation results. Firstly, the original image, the pulmonary vascular labeled image, and the lung parenchyma labeling result are executed by “AND” operation, and the results are used as the input for model training to obtain the pulmonary vascular segmentation model. Then, the original image, the pulmonary vascular labeled image, and the lung parenchyma segmentation result are executed by “AND” operation, and the result is used as the input for the model testing and the evaluation criteria. The overall flow is shown in Figure 2.

The leaky ReLU function in equation (5) is selected as the activation function instead of ReLU in the model, the sum of cross entropy and DICE coefficients in equation (2) is used as the final loss function, and Adam in equation (3) is used as the model optimizer.

(5) $$\begin{array}{c} f\left(x\right)=\max\left(0.01x,x\right) \end{array}$$

Because the training of 3D data is needed in the nnUnet network, the 2D slice data need to be integrated and converted into multiple sets of 3D nii.gz format data and grouped according to the training set, test set, and their respective corresponding label sets, which need to be corresponded one by one. Also, because the chest images are divided into CT and enhanced CT, i.e., CTA, the pulmonary vascular part is brighter in CTA than in CT, i.e., the pixel values are higher. Considering the effect of these pixel value changes on the pulmonary vascular segmentation, the CT and CTA data have to be trained separately.

## 3. Results and Discussion

The experimental data for this paper were obtained from the collaborating hospital, and a total of 67 sets of CT and CTA images were included in the data set. Among them, 24 sets of CT scans were acquired and reconstructed with the following parameters—slice layer thickness between 0.75 mm and 1.5 mm; voltage of 120 kVp; tube current of 88–215 mA; and slice number of 192 to 576.43 sets of CTA scans were acquired—and reconstructed with the following parameters—slice layer thickness between 0.625 mm and 1.5 mm; voltage of 120 kVp; tube current were 199 to 585 mA; and the number of slices was 285 to 557. Of these 67 data sets, 24 sets of CT data and 43 sets of CTA data were available. In order to reduce human interference, they were numbered and then divided completely randomly into two groups by random numbers: the training data set, containing 18 CT data sets and 34 CTA data sets, and the test data set, containing 6 CT data sets and 9 CTA data sets.

The hardware and software environment and equipment information required for the experiments are as follows: (1) CPU processor: Intel(R) Core(TM) i5-7500 CPU @ 3.40 GHz 3.40 GHz; (2) GPU processor: NVIDIA GeForce GTX 1080 Ti; (3) operating system: Windows 10 64 bit; (4) programming language and compilation environment: Python 3.7; PyCharm 2020.1 × 64.

A comparison experiment was performed between the two methods that combined the results of lung parenchymal segmentation and those that did not. The metrics used were DICE, undersegmentation rate (UR), and over-segmentation rate (OR), where UR and OR were calculated as follows:

(6) $$\begin{array}{c} OR=\frac{O}{R+O},\\ UR=\frac{U}{R+O}, \end{array}$$

where *R* is the number of target pixel points in the marker image, *O* is the number of pixel points that are not present in the marker image but are present in the target of the prediction result, and *U* indicates the number of pixel points that are present in the target of the marker image but are not present in the target of the prediction result.

The comparison of the evaluation criteria for the final results is shown in Tables 1 and 2. As can be seen in the tables, the average segmentation accuracy of the CT dataset improved from 81.7% to 83% and the CTA improved from 83% to 85%. This indicates that the segmentation of the pulmonary vasculature in combination with the segmentation of the lung parenchyma can effectively eliminate the influence of other tissues and obtain more accurate pulmonary vascular segmentation results.

Figures 3 and 4 show the segmentation results of pulmonary vessels in CT and CTA images, respectively, where (a) is ground truth, (b) is the corresponding 2D segmentation result, and (c) is the 3D segmentation result. From the results shown in the figure, it can be seen that nnUnet has a better segmentation effect on some boundary details and at the same time can effectively reduce the oversegmentation situation of the images.

In this paper, experiments were conducted on mainstream image processing methods such as Unet, Unet++, TransUnet, and Unet + Attention under the same experimental conditions. The experimental results were evaluated with DICE, OR, and UR, and the average values of each parameter are shown in Table 3.

From the above table, it can be seen that the method in this paper can produce better results on both CT and CTA images. The average accuracy is able to reach 84.2% and 87.7%, respectively, which is better than other methods and similar to the accuracy of Unet + Attention. It also outperforms other algorithms in terms of OR and UR. In addition, in this paper, six groups of CTs and nine groups of CTAs in the test group are exchanged with the data in the corresponding training group and the experiments are rerun for cross-validation purposes. The DICE coefficients obtained from the experiments are above 0.85, and the OR and UR coefficients are below 0.110. The accuracy of the algorithm in this paper can be verified.

## 4. Conclusions

In this paper, a deep learning-based approach was used for segmentation of pulmonary vessels, and improvements were made by combining pulmonary parenchymal segmentation with it. First, a lung parenchyma segmentation algorithm based on the Unet++ network model was designed and evaluated in several aspects. The algorithm was able to improve the evaluation metrics slightly even though more accurate results were obtained for the lung parenchyma segmentation task, indicating that the method is effective and accurate. Later, based on the obtained results for lung parenchyma segmentation, a nnUnet-based algorithm for lung vascular segmentation is designed, and the nnUnet model is studied. This method extracts image features from three dimensions, taking into account the extraction of global features and the underlying image details. Its application to the lung vessel segmentation task with the method studied in the previous chapters is implemented, and the same comparative experiments are performed, taking into account the differences between the lung vessel pixels in CT images and CTA images in the original data, respectively, to verify the accuracy of the algorithm.

The current method of segmentation of pulmonary vessels is mainly for the whole lung. In this paper, we combine lung parenchyma segmentation with pulmonary vessel segmentation to limit the segmentation area to the lung parenchyma region, avoiding the interference of excess impurities and improving the accuracy of segmentation.

## Figures and Tables

**Figure 1:** Model structure diagram.

**Figure 2:** Training and validation process.

**Figure 3:** CT image segmentation results: (a) ground truth; (b) 2D results; (c) 3D results.

**Figure 4:** CTA image segmentation results: (a) ground truth; (b) 2D results; (c) 3D results.

**Table 1:** Comparison of segmentation result indicators of CT data.

Indicator	Method	Dataset						Average
		1	2	3	4	5	6	
DICE	With pulmonary parenchyma	0.682	0.785	0.835	0.853	0.895	0.851	0.817
	Without pulmonary parenchyma	0.752	0.815	0.802	0.858	0.905	0.850	0.830
OR	With pulmonary parenchyma	0.446	0.144	0.083	0.148	0.135	0.061	0.169
	Without pulmonary parenchyma	0.346	0.133	0.085	0.128	0.093	0.065	0.142
UR	With pulmonary parenchyma	0.043	0.210	0.200	0.108	0.055	0.198	0.136
	Without pulmonary parenchyma	0.051	0.179	0.250	0.121	0.081	0.200	0.146

**Table 2:** Comparison of segmentation result indicators of CTA data.

Indicator	Method	Dataset									Average
		1	2	3	4	5	6	7	8	9	
DICE	With	0.82	0.83	0.80	0.76	0.81	0.90	0.89	0.79	0.84	0.83
	Without	0.85	0.82	0.85	0.82	0.80	0.90	0.89	0.84	0.91	0.85
OR	With	0.21	0.26	0.01	0.32	0.05	0.05	0.18	0.10	0.01	0.13
	Without	0.10	0.28	0.02	0.26	0.03	0.15	0.11	0.13	0.06	0.13
UR	With	0.10	0.03	0.33	0.06	0.27	0.13	0.02	0.25	0.26	0.16
	Without	0.15	0.23	0.24	0.05	0.29	0.05	0.09	0.14	0.10	0.15

**Table 3:** Comparison of average indexes of each segmentation method for CT and CTA images.

Indicator	Method	Datasets	
		CT	CTA
DICE	Unet	0.826	0.838
	Unet++	0.825	0.834
	TransUnet	0.805	0.815
	Unet + Attention	0.851	0.873
	nnUnet	0.842	0.877

OR	Unet	0.087	0.091
	Unet++	0.087	0.102
	TransUnet	0.080	0.089
	Unet + Attention	0.088	0.114
	nnUnet	0.079	0.105

UR	Unet	0.174	0.187
	Unet++	0.175	0.179
	TransUnet	0.200	0.223
	Unet + Attention	0.167	0.128
	nnUnet	0.119	0.110

## Data Availability

The data used to support the findings of this study are available from the corresponding author upon request.
